The article "Regulation of the Proliferation of Diabetic Vascular Endothelial Cells by Degrading Endothelial Cell Functional Genes with QKI-7" was published in 2022. Journal: Contrast Media Mol Imaging.

# Regulation of the Proliferation of Diabetic Vascular Endothelial Cells by Degrading Endothelial Cell Functional Genes with QKI-7

**DOI:** 10.1155/2022/6177809

**Published:** 2022-06-03

**Authors:** Jinmei Xu, Qingsong Zhao, Xu Han, Zheqi Zhang, Jiahui Qu, Zhifeng Cheng

**Affiliations:** Department of Endocrinology, the Fourth Affiliated Hospital of Harbin Medical University, Harbin 150001, Heilongjiang, China

## Abstract

**Background:**

Diabetes has emerged as one of the most serious and common chronic diseases of our times, causing life-threatening, disabling and costly complications, and reducing life expectancy. Studies have shown that cardiovascular morbidity is 1–3 times higher in diabetic patients than in normal people. There are many clinical and experimental data that prove that most of the complications of diabetes are related to atherosclerosis, which suggests that chronic hyperglycemia may induce an imbalance in the proliferation of vascular endothelial cells.

**Purpose:**

This study aims to explore the relationship between QKI-7 and vascular endothelial cell dysfunction and lay a foundation for further clarifying the molecular mechanism of endothelial cell damage in the process of diabetes with atherosclerosis.

**Methods:**

We chose blood samples and pluripotent stem cells and vascular endothelial cells of hospitalized patients with diabetes and diabetes atherosclerosis as research subjects. The expression levels of endothelial cell proliferation and genes related to endothelial cell proliferation were analyzed by RT-qPCR and Western blot, to study the influence of QKi-7 on the physiological state of endothelial cells. Through gene knockdown experiment, the effects of QKi-7 knockdown on functional genes and physiological functions of endothelial cells were analyzed. Finally, RNA immunoprecipitation was used to test the mutual effect among QKI-7 and the transcription level of functional genes, and the mRNA attenuation experiment proved that QKI-7 participated in the degradation process of functional genes.

**Results:**

The findings of the RT-qPCR and Western blot tests revealed that QKI-7 was highly expressed in blood samples of diabetic patients and atherosclerosis as well as in endothelial cells induced by human pluripotent stem cells and human vascular endothelial cells after high-glucose treatment. Overexpression and high glucose of QKI-7 resulted in inhibiting expressed function genes CD144, NLGN1, and TSG6 and upregulation of inflammatory factors TNF-*α*, IL-1*β*, and IFN-*γ*, leading to excessive proliferation of endothelial cells. After QKI-7 gene knockdown, the expression levels of CD144, NLGN1, and TSG6, inflammatory factors TNF-*α*, IL-1*β*, and IFN-*γ*, and the cell proliferation rate all returned to normal levels. RNA immunoprecipitation showed that QKi-7 interacted with CD144, NLGN1, and TSG6 mRNAs and was involved in the transcriptional degradation of functional genes through their interactions.

The article "Regulation of the Proliferation of Diabetic Vascular Endothelial Cells by Degrading Endothelial Cell Functional Genes with QKI-7" was published in 2022. Journal: Contrast Media Mol Imaging.

**Conclusion:**

This research initially revealed the relevant molecular mechanism of QKI-7 leading to the excessive proliferation of endothelial cells in diabetic and atherosclerotic patients. In view of the role of QKI-7 in diabetic vascular complications, we provided a potential target for clinical diabetes treatment strategies in the future.

## 1. Introduction

As of now, the number of people with diabetes exceeds 4 billion worldwide, and epidemiologists predict that the incidence of this disease will continue to rise, and deaths related to diabetes will double by 2030 [1]. Diabetes has emerged as one of the most serious and common chronic diseases of our times, causing life-threatening, disabling and costly complications, and reducing life expectancy [2]. Macrovascular complications such as coronary artery disease, stroke and peripheral artery disease, and microvascular complications such as retinopathy, nephropathy, and neuropathy are the major causes of high diabetes morbidity and mortality. Studies have shown that cardiovascular morbidity is 1–3 times higher in diabetic patients than in normal people [3]. Metabolic abnormalities associated with diabetes can lead to cardiovascular dysfunction, including chronic hyperglycemia, dyslipidemia, and insulin tolerance, which make the arteries prone to atherosclerosis. Diabetes changes the function of many cells, such as endothelial cells, smooth muscle cells, and platelets [4]. On the internal surface of blood vessels is a layer of endothelial cells, providing an active metabolical interface among tissues and blood, regulating blood flow, nutrient delivery, coagulation and thrombosis, and leukocyte exudation. The clinical correlation between diabetes and atherosclerosis has been well verified. There are many clinical and experimental data that prove that most of the complications of diabetes are related to atherosclerosis, which suggests that chronic hyperglycemia may induce an imbalance in the proliferation of vascular endothelial cells. The molecular mechanism between diabetes and atherosclerosis has not been elucidated, but the key process of endothelial activation in the process of vascular injury and atherosclerosis is due to the fine-tuning of many genes and transcription factors, such as the nuclear transcription factor NF-kB. NF-kB acts as an inflammatory mediator to regulate the entry point of the metabolic reaction. In the condition of high glucose, multiple inflammatory regulators can be activated by NK-kB, including tumor necrosis factor (TNF-*α*), IL-1B, IL-6, and protein kinase C (PKC) [5].

The article "Regulation of the Proliferation of Diabetic Vascular Endothelial Cells by Degrading Endothelial Cell Functional Genes with QKI-7" was published in 2022. Journal: Contrast Media Mol Imaging.

Endothelial cells can produce a variety of molecules related to vascular regulation and angiogenesis, and these molecules play important physiological regulatory roles at local or in distances [6]. Vascular endothelial cells (ECs) contribute to maintaining the integrity of blood vessels, regulating angiogenesis, inflammatory infiltration, monocyte adhesion, platelet aggregation, and intercellular barriers [7]. A major factor in the pathogenesis of vascular disease is changes in the vascular endothelium (such as atherosclerosis), and it is one of the key targets for preventing or slowing down the progression of vascular diseases [8]. Endothelial dysfunction is the first step in the atherosclerotic process. In the development of diabetes, vascular complications caused by vascular endothelial cell dysfunction will lead to increased monocyte adhesion, increased permeability, aberrant angiogenesis, increased thrombosis, and trends of blood flow disorders [9]. Quaking (QKI) proteins, as members of the RNA protein family, are involved in the pathogenesis of diabetic cardiomyopathy and atherosclerosis [10]. QKI proteins are members of the signal transduction and activation RNA family, which have relatively conservative SH2, SH3, and KH RNA-binding domains. Their main physiological function is to regulate the shearing of precursor RNA, mRNA nucleation, mRNA stability, protein translation, signal transduction, etc. [11]. Therefore, the research on endothelial cells has become a key and hot field of cardiovascular-related diseases, and the focus of many clinical studies has tended to explain the relationship between the changes in endothelial cell proliferation and the development of cardiovascular diseases.

According to relevant reports, the human genome encodes approximately 424 RNA-binding proteins (RBPs), and most RBPs are dysfunctional in the development of diabetes. The RNA-binding domains of RBPs are important regions for protein-recognizing RNA molecules. RBPs can combine precursor RNA5′ and 3′ UTR, intron and exon of the precursor RNA, and are entirely involved in the maturation, RNA localization, stability, and translation of precursor RNA [12]. Previous studies have shown that the 5′ cap structure and 3′ poly A tail structure of mRNA can be destroyed by decapping enzymes and adenosyltransferase, leading to their degradation. RBPs can lead to mRNA degradation by binding to the cis-activating element of mRNA and recruiting decapping enzymes and adenosyltransferase to mRNA [13].

The article "Regulation of the Proliferation of Diabetic Vascular Endothelial Cells by Degrading Endothelial Cell Functional Genes with QKI-7" was published in 2022. Journal: Contrast Media Mol Imaging.

There is a heterogeneous nucleic acid ribonucleoprotein k homology domain in QKI proteins, which is a part of Nova-1, Sam68, and a member of the FMRP family of KH RNA-binding proteins [14]. Based on the results available, QKI proteins mainly regulate the shearing of precursor mRNA, the export of mRNA, the stability of mRNA, and the translation of protein. At the same time, QKI proteins have a certain regulatory effect on apoptosis, cell cycle, and the development of glial cells [15]. The Kh domain of QKI-1 is wrapped in a large domain called GRP33-Sam68-GLD-1 (GSG) or activator of RNA signal transduction (STAR). Since QKI proteins play a huge role in the signal transduction pathway, this KH type of RNA-binding protein is also called RNA signal transduction activator protein [16]. All QKI homologs have unique GSG/STAR domains and unique RNA-binding capabilities. During embryonic development, QKI-5 has the highest expression abundance, while its expression in newborns has declined. The expressions of the other two homologs, QKI-6 and QKI-7, are in the late embryonic stage, and they express to the peak in the course of myelination [17]. It has been reported that the main transcription products of QKI include QKi-5, QKi-6, and QKi-7, which have relatively conservative sequences, and the different sequences mainly exist in the C-terminal. These three QKI allosteric proteins all existed in vascular endothelial cells, and QKI-5 has the highest expression abundance [18]. Both QKI-5 and QKI-6 have a favorable impact on angiogenesis, but they play a different role in different cell types, showing the key influence of the unique C-terminal sequence on its function. As for QKI-7, its C-terminal sequence is quite different from that of QKI-5 and QKI-6, but its effect on angiogenesis has not been clear yet [19].

Previously, researchers found that three major QKI family transcriptional isomers, QKi-5, QKi-6, and QKi-7, were all expressed in vascular endothelial cells, of which QKi-5 has the highest expression abundance. On the basis of available experiment data, human QKi-5 gene knockout leads to death in the embryo. Further investigations showed that QKI-5 knockout resulted in a remarkable reduction in the expression of pecam-1 and tie-2. Similarly, the knockout of QKI-5 also caused serious disturbances in the process of angiogenesis [20]. The latest research results showed that QKI-5 could significantly improve angiogenesis, and in lower limb ischemia animal models, QKI-5 could effectively increase the speed of blood flow recovery. Further studies also have shown that QKi-5 could bind to the 3′UTR of the STAT3 gene to stabilize its mRNA, and more stable RNA will promote the stability of VE-cadherin and the activation of VEGFR2 [21]. The research discovered that QKI-6 could promote the shear of HDAC7, which was beneficial to the differentiation of pluripotent stem cells into vascular smooth muscle cells. In an in vivo Matrigel experiment, QKi-6 and QKi-5 were overexpressed in vascular smooth muscle cells and endothelial cells. It was shown that the overexpression of both QKI-6 and QKI-7 significantly improved the formation of vascular structures, which further validated their promoting effect on angiogenesis [22]. Both QKI-5 and QKI-6 have a positive effect on angiogenesis; however, they differ in how they act and in what cell types they function. Through sequence alignment analysis, we found that their C-terminal sequence was less conservative, which could be inferred that its unique C-terminal structure had a great influence on its unique functional characteristics. QKi-7, QKi-5, and QKi-6 all belong to the QKI family, and the C-terminal sequence of QKi-7 is also significantly different from the other two. However, the effect of QKi-7 on vascular endothelial cell function proliferation in diabetic patients with arteriosclerosis remained unclear.

The article "Regulation of the Proliferation of Diabetic Vascular Endothelial Cells by Degrading Endothelial Cell Functional Genes with QKI-7" was published in 2022. Journal: Contrast Media Mol Imaging.

The findings show that the expression pattern of QKi-7 in diabetic patients with atherosclerosis was preliminarily investigated. The regulation function of QKi-7 on endothelial cell proliferation was elucidated. This research detected the high expression of QKi-7 in the blood samples of patients with diabetes mellitus complicated with atherosclerosis, and the same results were also obtained from HIPSC and VEC stimulated with a high concentration of glucose in vitro. Therefore, this study hopes to further explore what role QKI-7 plays in endothelial cells. We evaluated the changes in endothelial cell proliferation-related genes CD144, NLGN1, and TSG6 in hiPSCs with high-glucose treatment. Our research is to offer new theoretical profound understanding pathogenesis of diabetic atherosclerosis and provide a potential scheme for the clinical treatment of diabetic vascular complications. We selected blood samples and pluripotent stem cells and vascular endothelial cells of hospitalized patients with diabetes and diabetes atherosclerosis as research subjects. We used RNA immunoprecipitation to test the mutual effect among QKI-7 and the transcription level of functional genes, and the mRNA attenuation experiment proved that QKI-7 participated in the degradation process of functional genes.

## 2. Materials and Methods

### 2.1. Drugs and Instruments

PBS buffer was obtained from Biyuntian Biological Co., Ltd., China, Art. No.: C0221A. Streptozotocin was purchased from SIGMA Company, No.: S0130. Streptomycin was dissolved in PBS, prepared into 100 mg/mL of storage solution, filtered with a 0.22 *μ*m needle filter, and stored separately at −20°C. RNA extraction reagent TRIzol was purchased from Thermo Fisher Company, No.: 15596018. The reverse transcription kit was obtained from Takara Biological Co., Ltd., No.: RR037B. Fluorescence quantitative PCR reagents were purchased from Roche Company, No.: 4913850001. Both RIPA protein lysate and BCA protein concentration determination kit were obtained from Bibiyuntian Biological Co., Ltd., China, No.: P0013B. CD144-specific antibody was obtained from St. John's Laboratory, No.: STJ96234; NLGN1-specific antibody was purchased from Abcam, No.: ab153821. Anti-human-TNF-*α* was purchased from Cell Signaling Technology, Inc., No.:11948. IL-1*β*-specific antibody was purchased from CST, No.: 12703. IFN-*γ*-specific antibody was purchased from CST, No.: 8455. HRP-labeled goat anti-rabbit and goat anti-mouse secondary antibodies were purchased from Quanshijin Biotech Co., Ltd., Beijing, No.: HS101-01, HS201-01. PGI2 ELISA Kit was obtained from Elabscience Biological Co., Ltd., No.: E-EL-0022. Both L-glucose and D-glucose were purchased from SIGMA, No.: G5500, G7021. ECL protein chromogenic solution was purchased from Bio-Rad, No.: 1705060S. Human pluripotent stem cells were purchased from SIMGA, No.: IPSC0028. Human vascular endothelial cells were purchased from ATCC, No.: PCS-100-020. The kits of E-selection, ICAM-1, and VCAM-1 ELISA were purchased from R&D Biological Co., Ltd., No.: DSLE00, DCD540, DVC00. The remaining inorganic reagents were obtained from Xilong Science Co., Ltd. The full-wavelength microplate reader was obtained from Bio-Rad, USA, model: 450. The small desktop low-temperature refrigerated centrifuge was obtained from Thermo Fisher Company in the United States, model: 75002456. Western Blot electrophoresis and transfer instrument was obtained from Bio-Rad, USA, model: 1645050. A fluorescent quantitative PCR instrument was obtained from Bio-Rad, model: T100. The fluorescence quantitative PCR instrument was obtained from Thermo Fisher, model: QuantStudio 6. The chemiluminescence colorimeter was obtained from Bio-Rad, model: 1708265.

The article "Regulation of the Proliferation of Diabetic Vascular Endothelial Cells by Degrading Endothelial Cell Functional Genes with QKI-7" was published in 2022. Journal: Contrast Media Mol Imaging.

### 2.2. Clinical Samples

This study had been approved by the Fourth affiliated Hospital of Harbin Medical University ethics committee. All participants obtained the information orally or in writing and formally signed the informed consent. This study selects 120 type 2 diabetic patients in the Department of endocrinology from June 2018 to July 2020, and the inclusion and exclusion criteria were as follows. ①They should comply with the diagnostic criteria for T2DM in the 2017 edition of “Guidelines for the Prevention and Treatment of Type 2 Diabetes in China” [23]. The diagnostic criteria for T2DM are as follows: fasting blood glucos ≥7.0 mmol/L, postprandial blood glucose ≥11.1  mmol/L, or random blood glucose ≥ 11.1 mmol/L. T2DM can be diagnosed if one of the three conditions is met. ②The age of patients should be over or equal to 60. ③All patients undergo carotid artery examination with Doppler color ultrasound. ④There should be complete clinical data, and its exclusive criteria were as follows: excluding those with malignant tumors, secondary diabetes, gestational diabetes, acute and chronic infections of diabetes, peripheral arterial intervention, or surgical treatment, and those who do not cooperate with examinations or investigations, etc. Intima-media thickness (IMT) of the carotid artery was detected by color Doppler ultrasound in all patients. IMT<1.0 mm was considered normal, IMT 1.0～1.2 mm was considered an intimal thickening, and IMT>1.2 mm was considered plate formation. Plaque formation was determined according to whether the IMT value was >1.2 mm or local plaque formation, and all patients are divided into a diabetes and atherosclerosis group and a diabetes group. In addition, 60 cases of healthy gender- and age-matched examination persons were recruited. The inclusion criteria were as follows: ①fasting blood glucose≤6.1 mmol/L and 2 h postprandial blood glucose ≤7.8mmol/L; ②color Doppler ultrasound detection IMT <1.0 mm. The exclusion criteria were as follows: ①patients with malignant tumors, ②patients with peripheral arterial intervention or surgical treatment, ③patients with other systemic diseases, and ④those patients who do not cooperate with inspections or investigations.

Fasting venous blood was collected from each study subject. On the day of the blood sampling, the patient's detailed history was recorded and blood pressure was measured.

### 2.3. Cell Culture and Differentiation

Human vascular endothelial cells were cultured with 5 ng/ml rhVEGF, 5 ng/ml rhEGF, 5 ng/ml rhFGF basic, 15 ng/ml rhIGF-1, 10 mM L-glutamine, 0.75 U/ml HS, 1 *μ*g/ml hydrocortisone hemisuccinate, 50 *μ*g/ml ascorbic acid, and 2% FBS Vascular Cell Basal Medium.

Differentiation of human pluripotent stem cells was carried out as follows: human pluripotent stem cells were cultured in DMEM/F12 mixed medium, and N2, B27, 8 *μ*M CHIR99021, and 25 ng/ml BMP4 were added to the basic medium; after 3 days, the medium was replaced with StemPro 34 medium containing 200 ng/ml hVEGF and 2 *μ*M forskolin for 2 days; on the 6th day, CD144 positive cells were separated by magnetic bead separation and cultured in EGM-2 medium [24].

The article "Regulation of the Proliferation of Diabetic Vascular Endothelial Cells by Degrading Endothelial Cell Functional Genes with QKI-7" was published in 2022. Journal: Contrast Media Mol Imaging.

### 2.4. Glucose Treatment

Endothelial cells were plated at a density of 1105 cells/ml into 6-well cell culture plates, and D-glucose (5 mM, 50 mM) or L-glucose (Control, 50 mM) was added to the cell culture medium and incubated for 6 days. And the fresh cell culture medium supplemented with glucose was changed every 2 days.

### 2.5. CCK-8 Assay

The proliferation efficiency of endothelial cells in different treatment groups was measured at 0 h, 6 h, 24 h, 48 h, and 72 h, respectively. The instructions were strictly followed to perform the operation procedures. In a 24-well cell culture plate, 50 *μ*l CCK-8 solution was added to each well, and the cell-free well but with a cell culture medium was used as a negative control. The cells were cultured for 2 hours in a cell culture chamber, and the absorbance value at 450 nm was measured by spectrophotometer.

### 2.6. Overexpression of QKI-7

The QKI-7 sequence was cloned into the lentiviral vector pLVX-Puro to construct the pLVX-QKI-7-Puro expression plasmid, and pLVX-QKI-7-Puro was cotransfected with pspAX2 and pMD2.G into HEK-293T cells to obtain lentiviral culture medium expressing QKi-7.Cells overexpressing the QKi-7 gene could be obtained by infecting the harvested lentivirus with endothelial cells.

### 2.7. Fluorescence Quantitative PCR to Detect Gene Expression

Total cell RNA was extracted using the Trizol, and PrimeScript™ RT reagent Kit (Perfect Real Time) (RR037B, Takara) was used to reverse the transcription of RNA into cDNA. PCR instrument (T100, Bio-Rad) was used for cDNA synthesis, and the reaction conditions are 37°C for 15 min and 85°C for 5 s. According to TB Green® Fast qPCR Mix (4913850001, Roche) instructions, a qPCR reaction solution was prepared to test CD144, NLGN1, TSG6, TNF-*α*, IL-1*β*, and IFN-*γ*. The primer sequence of the internal reference gene GAPDH is shown in Table 1. The gene was amplified by a qPCR instrument (QuantStudio 6, Thermo Fisher). The RT-qPCR reaction program was predenaturation at 95°C for 30 s, PCR reaction at 95°C for 3 s, 60°C for 30 s, and cycle number 40.

### 2.8. Western Blot

1 × 10^7^ cells were mixed with 0.2 mL RIPA lysate with 2 *μ*l 100 *μ*M PMSF, After fully homogenizing, the slurry was placed on ice and cracked for 30 min, during which the cells were mixed with eddy oscillation once every 10 min. The supernatant was collected after centrifugation at 4°C for 12,000 g × 10 min, and the protein concentration was determined by the BCA method. The extracted total tissue protein was added with 5× loading buffer（v：*v* = 4 : 1） and then was bathed in boiling water for 5 min, followed by a Western blot test. After the transfer of the membrane, it was blocked in 5% BSA blocking solution at room temperature for 1 hour, and specific antibodies were used to detect CD144, NLGN1, TSG6, TNF-*α*, IL-1*β*, and IFN-*γ*, respectively, and were incubated overnight at 4°C (the working concentration of all antibodies is 1 : 1000, *v*:v dilution; the diluent is the blocking solution). After washing three times with TBST, the goat anti-mouse secondary antibody (working concentration: 1 : 5000) was used for incubation at room temperature for 1 h. Then, the ECL chemiluminescence kit was used for color development, and the images were taken by the Bio-Rad gel imaging system. The images were processed by Image Lab software, and GAPDH was used as an internal reference protein for quantitative analysis.

The article "Regulation of the Proliferation of Diabetic Vascular Endothelial Cells by Degrading Endothelial Cell Functional Genes with QKI-7" was published in 2022. Journal: Contrast Media Mol Imaging.

#### 2.8.1. ELISA Assay

The secretory expression level of E-selection, ICAM-1, VACM-1 in blood samples, and PGI2 in QKI-7 overexpressing cells were detected by a specific ELISA kit. The OD450 nm value was measured by a full-wavelength enzyme plate analyzer, and all operations were carried out in strict accordance with the actual instructions.

### 2.9. QKI-7 Knockdown

A total of 1 × 10^6^ endothelial cells were suspended into the Nucleofector buffer, and 5 *μ*M of QKi-7-specific siRNA was added to the suspension and then transferred to a 37°C biochemical incubator to continue incubating for 48 hours. The QKI-7 siRNA sequence is GUGAGAGAUUGGUAUUAGUU.

The mRNA and protein levels of CD144, NLGN1, TSG6, TNF-*α*, IL-1*β*, IFN-*γ,* and PGI2 were detected according to the above methods.

### 2.10. RNA-Binding Protein Immunoprecipitation

The RNA-binding protein immunoprecipitation test kit was purchased from Millipore (Art. No.: 17–700), and all the experimental steps were performed in accordance with the instructions [25]. The cell lysate was incubated with QKi-7-specific antibody and negative antibody IgG, the expressions of CD144, NLGN1, and TSG6 were detected by RT-qPCR after immunoprecipitation of RNA, and the results were evaluated by analyzing the relative gene expression levels of QKi-7 group and IgG group.

### 2.11. mRNA Attenuation Assay

The endothelial cells of overexpressing QKI-7 and the transcription inhibitor actinomycin D were coincubated for 0, 2, 4, 6, 8, and 12 hours, respectively, and the mRNA expression levels of CD144, NLGN1, and TSG6 in nonoverexpression cells and overexpression cells were used to evaluate the degradation function of QKI-7 for this gene [26].

### 2.12. Data Analysis

All statistical data were expressed as mean ± standard error (Mean ± SE). The differences between the experimental groups were analyzed by multiple comparison corrected analysis of variance or *t*-test to analyze the statistical significance (Primer 5, GraphPad Software). When *p* < 0.05, it indicated a statistically significant difference.

The article "Regulation of the Proliferation of Diabetic Vascular Endothelial Cells by Degrading Endothelial Cell Functional Genes with QKI-7" was published in 2022. Journal: Contrast Media Mol Imaging.

## 3. Results

### 3.1. QKI-7 Was Highly Expressed in the Blood of Diabetes and Atherosclerosis

QKI-5, QKI-6, and QKI-7 were all expressed in vascular endothelial cells, and both QKI-5 and QKI-6 were important factors in regulating angiogenesis. To explore the function of QKI-7 in the process of diabetes and atherosclerosis, we first tested the expression of QKI-7 in the blood samples of patients with diabetes and atherosclerosis. The findings proved that the expression of QKI-7 in the patients' blood of diabetes and atherosclerosis was significantly higher than its expression level in diabetic and normal samples (Figure 1(a)). It proved that the expression of QKI-7 was high in patients with diabetes and atherosclerosis. And the endothelial cell dysfunction markers E-selection, ICAM-1, and VCAM-1 showed an increasing trend in the normal group, the diabetic group, and the diabetic with atherosclerosis group (Figure 1(b)), which was consistent with the trend of QKi-7 among all groups.

### 3.2. QKI-7 Is Highly Expressed in Endothelial Cells Treated with High Glucose

To simulate the physiological state of endothelial cells in patients with diabetes and atherosclerosis in vitro, we took endothelial cells induced by anthropogenic pluripotent stem cells (hiPSCs) and commercial human vascular endothelial cells (VECs) as a model and treated both kinds of cells with different concentrations of glucose. It could be seen that Qki-7 was upregulated in a dose-dependent manner in high-glucose-treated human endothelial cells by RT-qPCR and WB (Figure 2). After human pluripotent stem cells were differentiated, different concentrations of glucose were used to treat endothelial cells and vascular endothelial cells, and the expression status of the QKI-7 gene in the transcription level and translation level was detected by RT-qPCR and western blot.

### 3.3. QKI-7 with High-Glucose Treatment Inhibited the Expression of CD144, NLGN1, and TSG6 in Endothelial Cells and Promoted Cell Proliferation

In order to detect whether the key genes of endothelial cells had changed after high-glucose treatment, we used RT-qPCR and western blot to detect the expression levels of transcription and translation of related genes of QKI-7 in hiPSCs after high-glucose treatment. The findings proved that the expression of CD144, NLGN1, and TSG6 in endothelial cells in the untreated group was significantly higher than that after high-glucose treatment (Figures 3(a) and 3(b)). Then, we tested the cell proliferation efficiency of different treatment groups through the CCK-8 experiments, and the results proved that the proliferation rate of hiPSC with high-glucose treatment was remarkably higher than the untreated group.

The article "Regulation of the Proliferation of Diabetic Vascular Endothelial Cells by Degrading Endothelial Cell Functional Genes with QKI-7" was published in 2022. Journal: Contrast Media Mol Imaging.

### 3.4. QKI-7 Significantly Inhibited the Expression of CD144, NLGN1, and TSG6 in Endothelial Cells

In order to verify the low expression of CD144, NLGN1, and TSG6 genes caused by the increased expression of QKI-7, we overexpressed the cells with QKI-7. Under the normal culture conditions, we detected the transcription level of key genes in the cells by RT-qPCR. The results showed that in the control group (Figure 4(b)) the mRNA of CD144, NLGN1, and TSG6 in QKi-7 was distinctly higher than that in overexpressed endothelial cells (Figure 4(a)). And western blot experiments also verified that the protein levels of these three genes were also lower than those of the control group (Figure 4(c)) while the proliferation rate of endothelial cells with QKI-7 overexpression was distinctly higher than that of the nonoverexpression group (Figure 4(d)).

### 3.5. QKI-7 Overexpression Promoted the Expression of Inflammatory Factors in Endothelial Cells

To verify if the promotion of endothelial cell proliferation by QKI-7 is also related to the abnormal expression of intracellular inflammatory factors, we detected the expression of TNF-*α*, IL-1*β,* and IFN-*γ* in hiPSC overexpression of QKI-7. The results showed that QKI-7 overexpression significantly increased the expression levels of TNF-*α*, IL-1*β*, and IFN-*γ* in endothelial cells (Figures 5(a) and 5(b)). The secretory expression level of the endothelial cell amplification marker molecule PGI2 was dramatically raised in the extracellular area, according to the ELISA data (Figure 5(c)).

### 3.6. CD144, NLGN1, and TSG6 Expression Levels Increased after QKI-7 Knockdown

The above tests proved that the expression of CD144, NLGN1, and TSG6 was inhibited in endothelial cells after high-glucose treatment and QKI-7 overexpression. In order to further verify whether this phenomenon is directly caused by the high expression of QKI-7, we knocked down the expression level of QKI-7 in hiPSC with high glucose by siRNA and detected the expression levels of CD144, NLGN1, and TSG6 in endothelial cells after a knockdown by RT-qPCR and western blot. As shown in the figure, after high-glucose treatment or with the QKI-7 gene knocked down (Figure 6(a)), the expression levels of CD144, NLGN1, and TSG6 were significantly increased (Figures 6(b) and 6(c)). And the proliferation efficiency of hiPSC with QKI-7 gene knockdown was distinctly lower than the control group (Figure 6(d)). Combined with the above results, it was suggested that the inhibition of key endothelial cell genes CD144, NLGN1, and TSG6 was caused by QKI-7, and it was further shown that QKI-7 had an important effect on the proliferation of endothelial cells. QKI-7-specific siRNA was used to knock down the QKI-7 gene in endothelial cells induced and differentiated by human pluripotent stem cells with high-glucose treatment;

The article "Regulation of the Proliferation of Diabetic Vascular Endothelial Cells by Degrading Endothelial Cell Functional Genes with QKI-7" was published in 2022. Journal: Contrast Media Mol Imaging.

### 3.7. QKI-7 Knockdown Inhibited the Expression of Inflammatory Factors TNF-*α*, IL-1*β*, and IFN-*γ*

The results of previous studies showed that the proliferation efficiency of QKI-7 overexpressed endothelial cells increased; the inflammatory factors TNF-*α*, IL-1*β*, and IFN-*γ* were expressed highly; the cell proliferation efficiency was significantly reduced after QKI-7 knockdown. In view of the relationship between inflammatory factors and cell proliferation, we speculated that TNF-*α*, IL-1*β*, and IFN-*γ* would also have corresponding changes in hiPSC after QKI-7 knockdown. In order to verify this conjecture, we used the specialty of siRNA to knock down the degree of QKi-7 gene expression in HIPSCs. The findings proved that the expression of inflammatory factors TNF*-α*, IL-1*β,* and IFN-*γ* was significantly reduced after QKi-7 knockdown (Figures 7(a) and 7(b)). The secretory expression of PGI2, a factor related to endothelial cell proliferation, was significantly reduced (Figure 7(c)), indicating that QKI-7 gene knockdown inhibited the proliferation of endothelial cells. Specific siRNA of QKI-7 was used to knock down the QKI-7 gene of endothelial cells after high-glucose treatment.

### 3.8. QKI-7 Specifically Binds to Key Endothelial Cell Genes CD144, NLGN1, and TSG6

This study found that there was a negative regulatory relationship between QKI-7 and key endothelial cell genes CD144, NLGN1, and TSG6, and QKI-7 was an RNA-binding protein. We speculated that the negative regulation of QKI-7 on CD144, NLGN1, and TSG6 was achieved through the interplay of QKI-7 with its mRNA. Therefore, we carried out RNA immunoprecipitation experiments, and the results showed that QKI-7 protein had significant specific binding with CD144, NLGN1, and TSG6 mRNA (Figure 8), compared with the negative control group. It showed that QKI-7 protein did specifically bind to the mRNAs of key genes CD144, NLGN1, and TSG6 through its RNA-binding protein properties and then regulated its expression. The QKI-7-specific antibody was used to carry out an RNA immunoprecipitation experiment in hiPSC after high sugar treatment, and the RNA product after QKI-7 coprecipitation was tested by RT-qPCR. ^*∗*^*p* < 0.05, taking the negative control IgG group as the control.

### 3.9. QKI-7 Promoted the Degradation of Key Genes CD144, NLGN1, and TSG6 at the Transcriptional Level

The above experimental findings proved that there was a close relationship between QKI-7 and the key genes of endothelial cells CD144, NLGN1, and TSG6 mRNAs, and QKI-7 had a negative regulatory effect on these 3 genes. Therefore, we speculated that the combination of the two promoted the degradation of key genes, which downregulated the transcription level in turn. To verify this conjecture, we treated endothelial cells of overexpressed QKI-7 with the transcription-suppressing compound actinomycin D. The results showed the degree of degradation of CD144, NLGN1, and TSG6 mRNAs in endothelial cells treated with actinomycin D was much lower than untreated group (Figure 9). The findings proved that QKi-7 bonded to CD144, NLGN1, and TSG6 mRNAs and promoted the degradation of their mRNAs, thereby affecting the physiological function of endothelial cells. In endothelial cells of overexpression QKI-7 (overexpression) and nonoverexpression (control), the contents of CD144, NLGN1, and TSG6 mRNA were detected at different times by RT-qPCR after actinomycin D treatment.

The article "Regulation of the Proliferation of Diabetic Vascular Endothelial Cells by Degrading Endothelial Cell Functional Genes with QKI-7" was published in 2022. Journal: Contrast Media Mol Imaging.

## 4. Discussion

Diabetes has emerged as one of the most serious and common chronic diseases of our times, causing life-threatening, disabling and costly complications, and reducing life expectancy [2]. The global prevalence of diabetes had reached pandemic proportions with the 9th edition of the IDF reporting a prevalence of 9% (463 million adults) in 2019. The rising prevalence of diabetes has been attributed principally to the aging of populations [27]. There are many clinical and experimental data that prove that most of the complications of diabetes are related to atherosclerosis, which suggests that chronic hyperglycemia may induce an imbalance in the proliferation of vascular endothelial cells. In this investigation, the expression of QKI-7 in clinical blood samples of diabetic patients with atheroma was significantly higher than its expression level in samples from simple diabetic patients and normal people. And by detecting the expression levels of the markers E-selection, ICAM-1, and VCAM-1 related to the progression of type 2 diabetes, we found that the expression levels of these three markers in patients with diabetes and atherosclerosis were much higher than those of people with simple diabetes or healthy individuals. It showed that the high expression of QKI-7 had a certain relationship with the severity of diabetes. And in the endothelial cells after differentiated human pluripotent stem cells and human vascular endothelial cells, we found that a high concentration of glucose treatment dramatically elevated the expression of QKI-7. Therefore, in the following mechanism discussion, endothelial cells (HIPSCs) induced by human pluripotent stem cells and human vascular endothelial cells (VECs) can be used as experimental models.

The article "Regulation of the Proliferation of Diabetic Vascular Endothelial Cells by Degrading Endothelial Cell Functional Genes with QKI-7" was published in 2022. Journal: Contrast Media Mol Imaging.

It has been reported that the main transcription products of QKI include QKi-5, QKi-6, and QKi-7, which have relatively conservative sequences, and the different sequences mainly exist in the C-terminal. These three QKI allosteric proteins all existed in vascular endothelial cells, and QKI-5 has the highest expression abundance [18]. Both QKI-5 and QKI-6 have a favorable impact on angiogenesis, but they play a different role in different cell types, showing the key influence of the unique C-terminal sequence on its function. As for QKI-7, its C-terminal sequence is quite different from that of QKI-5 and QKI-6, but its effect on angiogenesis has not been clear yet [19].

Among the genes related to the proliferation of endothelial cells, CD144 is an important marker of endothelial cells, which is extremely important for the integrity of blood vessel walls and angiogenesis [28]. NLGN1 is a cell surface protein, and recent research has revealed that NLGN1 also has a significant impact on the process of angiogenesis. The results of in vitro experiments show that the expression of NLGN1 is high in vascular endothelial cells, and its expression dynamics have a significant impact on the formation of endothelial cell vascular walls.

In studies about the complications of type 1 diabetes, the expression of TNF-*α* in the plasma of patients with proliferative retinopathy is remarkably increased. The cooperation of IL-1*β* and TNF-*α* can jointly promote angiogenesis, and the two can not only promote the synthesis of collagen but also stimulate the activity of glial cells and fibroblasts and promote cell proliferation [29]. Researchers also discovered that a lipid molecule called cycloprostaglandin (PGI2) can reflect the link between cardiovascular proliferation and vascular damage by affecting cell expansion, cell adhesion, permeability, and vascular tone. According to available reports, PGI2 is derived from arachidonic acid metabolites and can be continuously secreted and expressed by endothelial cells. The results of in vivo experiments show that knockout of NLGN1 results in the failure of vascular bundle formation [30]. TSG6 is a TNF-*α*/IL-1 inducible secreted protein with a hyaluronic acid-binding domain, which significantly alters the formation of ECM by disrupting the link between TSG6 and hyaluronic acid by specific antibodies. In a human model of diabetes, subconjunctival injection of recombinant TSG6 protein can promote the repair of corneal epithelial cells by activating primary progenitor cells and accelerating the polarization of M2 macrophages [31]. It is usually regarded as the main regulator of blood vessels. When endothelial cells proliferate rapidly, the secretory expression of PGI2 will increase significantly [32]. In previous studies, researchers had found that in patients who have type 2 diabetes or atherosclerosis, the excessive proliferation of endothelial cells was associated with excessive secretion of PGI2.

The article "Regulation of the Proliferation of Diabetic Vascular Endothelial Cells by Degrading Endothelial Cell Functional Genes with QKI-7" was published in 2022. Journal: Contrast Media Mol Imaging.

Both QKI-5 and QKI-6 have a positive effect on angiogenesis; however, they differ in how they act and in what cell types they function. Through sequence alignment analysis, we found that their C-terminal sequence was less conservative, which could be inferred that its unique C-terminal structure had a great influence on its unique functional characteristics. QKi-7, QKi-5, and QKi-6 all belong to the QKI family, and the C-terminal sequence of QKi-7 is also significantly different from the other two. However, the effect of QKi-7 on vascular endothelial cell function proliferation in diabetic patients with arteriosclerosis remained unclear. This research detected the high expression of QKi-7 in the blood samples of patients with diabetes mellitus complicated with atherosclerosis, and the same results were also obtained from HIPSC and VEC stimulated with a high concentration of glucose in vitro. Therefore, this study hopes to further explore what role QKI-7 plays in endothelial cells. We evaluated the changes in endothelial cell proliferation-related genes CD144, NLGN1, and TSG6 in hiPSCs with high-glucose treatment. The findings revealed that the expressions of CD144, NLGN1, and TSG6 in the group with high-glucose treatment were remarkably significantly lower than those of the control group, while the CCK-8 experimental results showed that the proliferation efficiency of hiPSC was abnormally increased after high-glucose treatment. In order to determine that the above phenomenon was directly caused by the changes in the expression of QKI-7, we tested the expression changes of the key factors of human endothelial cell CD144, NLGN1, and TSG6 in the overexpression of QKI-7 in hiPSCs. The findings revealed that the expressions of the three key factors in the overexpression of QKI-7 in hiPSCs were significantly reduced. In order to further clarify whether the proliferation ability of endothelial cells was damaged, we tested the expression level of cytokines related to endothelial cell proliferation, and the findings revealed that the levels of TNF-*α*, IL-1*β*, and IFN-*γ* in the overexpression of QKI-7 in hiPSCs were remarkably higher than those in normal endothelial cells, and the secretion level of endothelial cell proliferation-related molecules PGI2 in the overexpression of QKI-7 in hiPSCs was significantly increased. It further suggested the rapid proliferation state of endothelial cells when QKI-7 was highly expressed, and the results of CCK-8 finally showed that the overexpression of QKI-7 led to a significant increase in cell proliferation efficiency. It showed that QKI-7 overexpression had a remarkable stimulating effect on endothelial cell development, which was also consistent with the endothelial cell proliferation observed in patients with diabetes and atherosclerosis in the clinic [33]. In further research, we also found that after knocking down the QKI-7 expression level in hiPSC by siRNA, the expression levels of key endothelial cell genes CD144, NLGN1, and TSG6 were significantly increased; the expression of endothelial cell proliferation-related cytokine TNF -*α*, IL-1*β*, IFN-*γ*, and PGI2 also decreased; the proliferation efficiency of endothelial cells was significantly reduced. Based on the above results, we can speculate that QKI-7 has a significant impact on the proliferation of endothelial cells.

The article "Regulation of the Proliferation of Diabetic Vascular Endothelial Cells by Degrading Endothelial Cell Functional Genes with QKI-7" was published in 2022. Journal: Contrast Media Mol Imaging.

## 5. Conclusion

There are many clinical and experimental data that prove that most of the complications of diabetes are related to atherosclerosis, which suggests that chronic hyperglycemia may induce an imbalance in the proliferation of vascular endothelial cells. To clarify the molecular mechanism of QKI-7 leading to the excessive proliferation of endothelial cells in diabetes and atherosclerosis, We analyzed the function of QKI-7 under physiological conditions. Relevant literature indicated that QKI-7, one of the RNA-binding protein families, might bind specific mRNA and recruit decapping enzyme and adenylyltransferase to target mRNA, leading to the destruction of its 5′cap structure and ultimately destroying the stability of the target mRNA, which would cause its degradation [34]. In view of these findings, combined with the previous results of this study, the overexpression of QKI-7 reduced the expression levels of key genes CD144, NLGN1, and TSG6 in endothelial cells. We speculated that QKI-7 might interact with these three key genes in endothelial cells at the transcriptional level and caused the degradation of its transcription products. Therefore, we carried out RNA immunoprecipitation experiments in endothelial cells. The results showed that QKI-7 could directly bind to the mRNA of the key factors of endothelial cells CD144, NLGN1, and TSG6, which was consistent with the characteristics of QKI-7's RNA-binding protein. At the same time, the results of mRNA stability experiments showed that after QKI-7 was combined with CD144, NLGN1, and TSG6 mRNA, it significantly reduced RNA stability and accelerated the degradation of CD144, NLGN1, and TSG6 mRNA levels, which resulted in an imbalance in endothelial cell proliferation.

The article "Regulation of the Proliferation of Diabetic Vascular Endothelial Cells by Degrading Endothelial Cell Functional Genes with QKI-7" was published in 2022. Journal: Contrast Media Mol Imaging.

In summary, this study initially revealed the relevant molecular mechanism of QKI-7 leading to the excessive proliferation of endothelial cells in diabetic and atherosclerotic patients. In view of the role of QKI-7 in diabetic vascular complications, we provided a potential target for clinical diabetes treatment strategies in the future. Our future research direction is to combine QKI-7 with the clinical treatment of diabetes.

## Figures and Tables

**Figure 1:** QKI-7 was highly expressed in patients with diabetes and atherosclerosis. ^*∗*^*p* < 0.05, taking the normal patient group as the control. From clinical blood samples of normal patients, diabetic patients, and diabetic patients with atherosclerosis, the expression level of QKI-7 was detected by RT-qPCR (a) and the ELISA (b) assay to detect the secretory expression level of endothelial cell dysfunction markers E-selection, ICAM-1, and VCAM-1 in blood samples.

**Figure 2:** High concentration of glucose induced the upregulation of the QKI-7 gene. ^*∗*^*p* < 0.05, with the untreated group as the control.

**Figure 3:** QKI-7 with high-glucose treatment inhibited the expression of CD144, NLGN1, and TSG6 in endothelial cells and promoted cell proliferation. ^*∗*^*p* < 0.05, with the untreated group as the control. Treated endothelial cells induced by differentiation of human pluripotent stem cells with 50 mM high concentration glucose, and detection of the expression levels of CD144, NLGN1, and TSG6 by RT-qPCR (a) and western blot (b). CCK-8 was used to evaluate the changes in cell proliferation efficiency of the high-glycemic treatment group and the untreated group (c).

**Figure 4:** The effect of QKI-7 overexpression on endothelial cell functional genes and proliferation efficiency QKI-7 was overexpressed in endothelial cells induced by human pluripotent stem cells (a), which significantly reduced the transcription level (b) and translation level (c) of CD144, NLGN1, and TSG6 and promoted the proliferation of endothelial cells (d). ^*∗*^*p* < 0.05, with the untreated group as the control.

**Figure 5:** QKI-7 overexpression increased the expression levels of inflammatory factors of TNF-*α*, IL-1*β*, and IFN-*γ*.^*∗*^*p* < 0.05, with the untreated group as the control. The overexpression of QKI-7 in endothelial cells induced by human pluripotent stem cells significantly increased the transcription level (a) and translation level (b) of the cytokines TNF-*α*, IL-1*β*, and IFN-*γ*. ELISA results showed that the extracellular secretion level of PGI2 rose noticeably (c).

The article "Regulation of the Proliferation of Diabetic Vascular Endothelial Cells by Degrading Endothelial Cell Functional Genes with QKI-7" was published in 2022. Journal: Contrast Media Mol Imaging.

**Figure 6:** QKI-7 knockdown significantly increased the expression of CD144, NLGN1, and TSG6 and reduced cell proliferation efficiency.^*∗*^*p* < 0.05, with the nonknockdown group as control. RT-qPCR (a, b) and western blot (c) detected the transcription and translation levels of key endothelial cell genes QKI-7, CD144, NLGN1, and TSG6; the CCK-8 experiment detected the change in cell proliferation efficiency (d).

**Figure 7:** QKI-7 knockdown promoted cell proliferation ^*∗*^*p* < 0.05, with the nonknockdown group as the control. The transcription and translation levels of cytokines TNF-*α*, IL-1*β,* and IFN-*γ* were detected by RT-qPCR (a) and western blot (b), respectively. At the same time, ELISA detected the secretory expression of cell proliferation-related factor PGI2 (c).

**Figure 8:** The interaction between QKI-7 protein and CD144, NLGN1, and TSG6 mRNA.

**Figure 9:** QKI-7 promotes the degradation of CD144, NLGN1, and TSG6 genes at the transcriptional level ^*∗*^*p* < 0.05, taking the negative control DMSO group as the control.

**Table 1:** Primers for RT-qPCR.

Primers	Sequence
CD144-F	AAACACCTCACTTCCCCATC
CD144-R	ACCTTGCCCACATATTCTCC
NLGN1-F	ATGATGGAAGTGTCTTGGCAAGTT
NLGN1-R	CTTTGCAGCCTGATCGCCTGTA
TSG6-F	TCACCTACGCAGAAGCTAAGGC
TSG6-R	TCCAACTCTGCCCTTAGCCATC
TNF-*α*-F	ATGGCATGGACTGTGGTCATGAGT
TNF-*α*-R	ATGGCATGGACTGTGGTCATGAGT
IL-1*β*-F	CCACAGACCTTCCAGGAGAATG
IL-1*β*-R	GTGCAGTTCAGTGATCGTACAGG
IFN-*γ*-F	TTCTTACAACACAAAATCAAATCT
IFN-*γ*-R	TTCTTACAACACAAAATCAAATCA
GAPDH-F	CATGTTCGTCATGGGTGTGAACCA
GAPDH-R	ATGGCATGGACTGTGGTCATGAGT

## Data Availability

The datasets used and/or analyzed during the current study are available from the corresponding author on reasonable request.
